The article "Relationship between Peripheral Blood miR-181c, miR-101, and Cognitive Impairment in Patients with Diabetes Mellitus Complicated with Acute Stroke" was retracted in 2024. Reasons: signs of a paper mill; suspected computer-generated content; unreliable results or conclusions; lack of ethics approval or compliance.

# Relationship between Peripheral Blood miR-181c, miR-101, and Cognitive Impairment in Patients with Diabetes Mellitus Complicated with Acute Stroke

**DOI:** 10.1155/2022/5777106

**Published:** 2022-09-30

**Authors:** Mengxian Shu, Chunhui Xiang

**Affiliations:** ^1^Department of Pulmonary Disease Diabetes Mellitus, The Central Hospital of Enshi Autonomous Prefecture, Enshi, Hubei 445000, China; ^2^Department of Neurosurgery, The Central Hospital of Enshi Autonomous Prefecture, Enshi, Hubei 445000, China

## Abstract

**Objectives:**

To explore the relationship between peripheral blood microRNA-181c (miR-181c), microRNA-101 (miR-101), and cognitive impairment (CI) in patients with diabetes mellitus (DM) complicated with acute stroke (AS).

**Methods:**

A retrospective analysis was performed on 70 patients with DM complicated with AS admitted to the hospital between January 2019 and December 2021. According to presence or absence of CI, they were divided into CI group (41 cases) and non-CI group (29 cases). The clinical characteristics and general data (blood glucose and blood lipid) of patients were statistically analyzed. The relative expression levels of miR-181c and miR-101 in peripheral blood were detected by real-time fluorescence quantitative PCR. The risk factors of CI were analyzed by logistic regression analysis. The diagnostic value of peripheral blood miR-181c and miR-101 for CI was evaluated by receiver operating characteristic (ROC) curves.

**Results:**

The relative expression levels of peripheral blood miR-181c and miR-101 in the CI group were lower than those in the non-CI group (*P* < 0.05). The occurrence of CI was related to age, course of DM, AS location, time from onset to admission, HbA1c, TG, UA, and Hcy levels (*P* < 0.05). Logistic regression analysis showed that age, AS location, HbA1c, miR-181c, and miR-101 were related influencing factors of CI in patients with DM complicated with AS (*P* < 0.05). The results of ROC curves analysis showed that AUC, sensitivity, and specificity of miR-181c combined with miR-101 for predicting CI were 0.865, 73.17%, and 89.66%, respectively (*P* < 0.05).

**Conclusions:**

The peripheral blood miR-181c and miR-101 are low expressed in patients with DM complicated with AS, and advanced age, intracortical AS lesions, increased HbA1c, and low expression of miR-181c and miR-101 are all independent risk factors for CI in patients with DM complicated with AS. Besides, the combined detection of miR-181c and miR-101 expression has a good diagnostic value for CI.

## 1. Introduction

Diabetes mellitus (DM) is a glucose, lipid, and protein metabolic disorder syndrome caused by genetic, immune disorders, microbial infection, and other pathogenic factors, which can lead to increased cholesterol levels, decreased red blood cell deformability, and hypercoagulable state of organism, and promote thrombosis, thus easily inducing the occurrence of acute stroke (AS) [1, 2]. Some studies have found that DM microvascular complications are a high-risk factor for cognitive impairment (CI), which can cause neuronal degeneration and induce CI by inhibiting the insulin post-transport receptor signaling pathway, which has a serious impact on the work and life of patients [3, 4]. In recent years, microRNAs (miRNAs), which are widely present in brain tissue and have a regulatory effect on post-transcriptional protein expression, have become a research hotspot for their roles in neurogenesis, angiogenesis, and other cell biology [5]. MicroRNA-181c (miR-181c) is a member of the miR-181 family, and its overexpression increases reactive oxygen species production and affects mitochondrial genome protein coding [6]. Micro RNA-101 (miR-101) is sensitive to hypoxia, participates in cellular amino acid response, and plays an important regulatory role in neural tissue [7]. Previous studies have reported the changes of serum miR-181c levels in patients with acute cerebral infarction and the protective effect of miR-101 on cerebral ischemia-reperfusion injury, but there are relatively few studies reporting the changes of miR-181c and miR-101 levels in peripheral blood of patients with DM complicated with AS [8]. In addition, there is also a lack of research on the correlation between serum miR-181c and miR-101 levels and CI degree in patients with DM complicated with AS. In order to provide a molecular biological reference index for the prediction of cognitive dysfunction and early intervention planning in diabetes and patients, this study analyzed the relationship between the levels of miR-181c and miR-101 in peripheral blood and CI degree in patients with DM complicated with AS and the predictive value of the two on CI occurrence.

## 2. Materials and Methods

### 2.1. General Information

A retrospective analysis of 70 patients with DM complicated with AS admitted to our hospital from January 2019 to December 2021 was performed. Inclusion criteria were as follows: patient has a history of DM [9], patient met the diagnostic criteria for AS (the patient developed acute symptoms such as limb numbness and decreased muscle strength, and the appearance of cerebral infarction was confirmed by cranial CT or magnetic resonance imaging) and was admitted within 48 hours of developing AS [10], and patient's clinical medical records are complete. Exclusion criteria were as follows: patients with severe organ dysfunction or malignant tumor; patients with combined craniocerebral trauma, cerebrovascular malformation, or cerebral hemorrhage; patients with previous cognitive dysfunction; and patients with acute and chronic infectious diseases in various tissues and organs of the body. The patients were divided into 41 cases in the CI group and 29 cases in the non-CI group according to whether CI occurred or not, and the diagnosis [11] of CI was made by combining diagnostic criteria from the authoritative literature, the patient's history, physical examination and cognitive screening results.,

### 2.2. Methods

#### 2.2.1. Clinical Information Collection

The general data of the included subjects were collected through the hospital electronic medical record system, including gender, age, education level, body mass index (BMI), combined underlying diseases (hypertension and coronary heart disease), smoking history, drinking history, DM duration, AS location (subtentorial, subcutaneous, and cortical), type of AS, time from onset to admission, National Institute of Health Stroke Scale (NIHSS) score, fasting blood glucose (FBG), glycated hemoglobin (HbA1c), triacylglycerol (TG), total cholesterol (TC), low-density lipoprotein cholesterol (LDL-C), high-density lipoprotein cholesterol (HDL-C), total bilirubin (TBIL), direct bilirubin (DBIL), uric acid (UA), homocysteine (Hcy), thyroid-stimulating hormone (TSH)), and cysteine (Cys).

#### 2.2.2. Detection of miR-181 and miR-101 Expression in Peripheral Blood

In the morning of the next day after admission, 5 mL of fasting venous blood was collected from all the included subjects through the cubital vein and then anticoagulated and stored at low temperature. Total RNA was extracted by adding TRIzol and reverse transcribed into cDNA. miR-181c and miR-101 with cDNA as template were amplified, and PCR was used to perform fluorescence quantitative PCR reaction. The reaction conditions are as follows: 3 replicate wells for all samples, 95°C for 15 min, 94°C for 15 s, 60°C for 35 s, repeated 40 times. Using U6 as the internal reference, primer sequences are as follows: miR-181c upstream 5′-AACAUUCAACCUGUCGGUGAGU-3′, downstream 5′-UCACCGACAGGUUGAAUGUUUU-3′; miR-101 upstream 5′-CGTGCCAGACATGGACCTAT-3′, downstream 5′-CGGGGTAGGTGAAGACGAAG-3′; U6 upstream 5′-TCAGTTTGCTGCTGTTCTGGGTG-3′, downstream 5′-GGGTTGGCTGGAAAGGA-3′. The relative expression levels of miR-181c and miR-101 were calculated by 2-△△CT method. All steps were carried out in strict accordance with the instructions of each instrument and reagent.

### 2.3. Statistical Processing

SPSS 22.0 statistical software was used for data analysis, measurement data were expressed by ($\bar{x}\pm s$), differences between groups were expressed by two-sample independent *t*-test, count data were expressed by rate, and differences between groups were expressed by *χ*2 test. Univariate analysis and binary logistic regression were used to analyze the risk factors for the occurrence of CI in patients with DM complicated with AS. The receiver operator characteristic curve (ROC) was used to detect the diagnostic value of miR-181c and miR-101 expression in peripheral blood for the occurrence of CI in patients with DM complicated with AS. Two-sided *P* < 0.05 was considered to be statistically significant.

## 3. Results

### 3.1. Comparison of Relative Expression Levels of miR-181c and miR-101 in Peripheral Blood of Patients with DM Complicated with AS in the CI Group and the Non-CI Group

The relative expressions of miR-181c and miR-101 in peripheral blood of patients with DM complicated with AS in the CI group were significantly lower than those in the non-CI group (*t* = 8.534, 14.279, *P* < 0.05), as shown in Figure 1.

### 3.2. Univariate Analysis  of  CI in Patients with DM Combined with AS

The occurrence of CI in patients with DM combined with AS was related to age, duration of DM, AS location, time from onset to admission, and levels of HbA1c, TG, UA, and Hcy (*P* < 0.05). There was no relationship with gender, education level, BMI, underlying disease, smoking history, drinking history, duration of DM, AS type, NIHSS score, and FBG, TC, LDL-C, HDL-C, TBIL, DBIL, TSH, and Cys levels (*P* > 0.05), as shown in Figure 2 and Table 1.

### 3.3. Logistic Regression Analysis Affecting the Occurrence of CI in Patients with DM Complicated with AS

The difference variables that affected the cognitive function of patients with DM and AS were assigned and divided according to the mean value of all patients as the critical value, and the detection level was *α* = 0.05. The assignments of dependent and independent variables are shown in Table 2. Logistic regression analysis showed that age (OR = 2.784, *P*=0.038), AS location (OR = 2.697, *P*=0.024), HbA1c (OR = 2.751, *P*=0.031), miR-181c (OR = 2.759, *P*=0.024) = 0.032), and miR-101 (OR = 2.702, *P*=0.047) were related factors affecting the occurrence of CI in patients with DM complicated with AS, as shown in Table 2.

### 3.4. The Diagnostic Value of miR-181c and miR-101 Expression in Peripheral Blood for CI in Patients with DM Complicated with AS

The ROC Table 3 results showed that the AUC of miR-181c and miR-101 in peripheral blood for predicting the occurrence of CI in patients with DM complicated with AS was 0.816 and 0.783, respectively, and the cutoff values were 0.91 and 1.01, respectively. Combined detection was used to predict the area under the curve of CI in patients with DM complicated with AS (area under curve, AUC) which was 0.865, and the sensitivity and specificity were 73.17% and 89.66%, respectively (*P* < 0.05), as shown in Figure 3 and Table 4.

## 4. Discussions

DM patients often suffer from AS and other acute complications due to endocrine disorders, glycolipoprotein metabolism imbalance, and microvascular disease. Some studies have found that more than half of DM patients with AS can have CI, which seriously affects their quality of life [12, 13]. Therefore, finding simple and noninvasive biomarkers for early screening and diagnosis of cognitive impairment in DM patients with AS is of great significance to the clinical health management of DM patients. miRNA is a key regulatory molecule that plays an important role in the development and function of the nervous system [14]. This study mainly explored the relationship between the expression of miR-181c and miR-101 in peripheral blood and CI occurrence in patients with DM complicated with AS.

The results of this study showed that the relative expressions of miR-181c and miR-101 in the peripheral blood of patients with DM combined with AS in the CI group were significantly lower than those in the non-CI group, indicating that the expressions of miR-181c and miR-101 in peripheral blood of patients with DM complicated with AS were downregulated, which might lead to the occurrence of CI. Studies by Lian et al. [15] and others found that CI was related to neuronal apoptosis and mitochondrial dysfunction, and studies by Meng et al. [16] found that miR-181c was downregulated in AS patients. MiR-181c is an miRNA widely expressed in the central nervous system, and it is often abnormally expressed in a variety of neurodegenerative and neuropsychiatric diseases with cognitive deficits. The abnormal expression of miR-181c can participate in the regulation of neuronal function by regulating mitochondrial histone coding [17]. The hippocampus is the key and basis for the formation of long-term memory and is closely related to cognitive functions such as learning and memory. miR-101 is extremely sensitive to hypoxia and highly expressed in synapses, and it participates in the proliferation and apoptosis of hippocampal neurons by negatively regulating the degradation of amyloid precursor in hippocampal neurons, and thus plays a neuroprotective role. miR-101 may participate in the regulation of hippocampal neuron apoptosis and regeneration through endogenous antioxidant pathways, affecting synaptic function and structure, and then regulating cognitive function in patients [18].

The results of this study showed that the occurrence of CI in patients with DM combined with AS was related to age, duration of DM, AS location, time from onset to admission, and levels of HbA1c, TG, UA, and Hcy, similar to the results of other studies, suggesting that cognitive function in patients with DM combined with AS may be related to factors such as age, duration of disease, damage to cerebral cortex, treatment delay, blood sugar control, and blood lipid level. Further multiple linear regression analysis was used to analyze the influencing factors of cognitive function in patients with DM complicated with AS. The results showed that age, AS location, HbA1c, miR-181c, and miR-101 were independent influencing factors on cognitive function of DM patients with AS, which indicated that the elderly, high HbA1c level, cortex, miR-181c, and miR-101 expression level were more likely to have CI. Elderly patients are often accompanied by decreased cerebral cortical cells and decreased cerebral perfusion, which increase the risk of CI. Cognitive function is generated and maintained in the complex system network of the brain. Current research generally believes that the brain functional area of cognitive function is located in the cerebral cortex, and the cerebral cortex damage is most closely related to CI in the site of AS occurrence [19]. The level of HbA1c reflects the glycemic control of patients. The toxic effect of hyperglycemia on the brain tissue of AS patients can lead to severe cerebral ischemia and hypoxia, which significantly increases the risk of CI [20]. miR-181c and miR-101 are involved in the occurrence and development of CI by regulating mitochondrial gene histone coding and neuronal apoptosis in the hippocampus in patients with DM combined with AS [6, 20]. In this study, ROC curve was used to evaluate the diagnostic value of peripheral blood miR-181c and miR-101 expression for CI in patients with DM complicated with AS. The results showed that the AUC of miR-181c and miR-101 in peripheral blood for predicting the occurrence of CI in patients with DM complicated with AS was 0.816 and 0.783, respectively. The AUC of combined detection for predicting the occurrence of CI in patients with DM complicated with AS was 0.865, with a sensitivity and specificity of 73.17% and 89.66%, respectively. This indicates that the combined detection of miR-181c and miR-101 in peripheral blood has high specificity in diagnosing the occurrence of CI in patients with DM complicated with AS and has the best diagnostic performance for CI. It suggested that the abnormal expression of miR-181c and miR-101 in peripheral blood could be used as a reliable indicator for predicting the occurrence of CI in patients with DM complicated with AS.

In conclusion, advanced age, intracortical AS lesions, increased HbA1c, and low expression of miR-181c and miR-101 are all independent risk factors for CI in patients with DM complicated with AS. Besides, the combined detection of miR-181c and miR-101 expression in peripheral blood has a good diagnostic value for CI in patients with DM complicated with AS. The disadvantage of this study is that the number of selected samples is limited, and the correlation between the severity of CI and the expression of miR-181c and miR-101 in patients with DM complicated with AS has not been compared and analyzed.

## Figures and Tables

**Figure 1:** Comparison on relative expression levels of peripheral blood miR-181c and miR-101 between the CI group and the non-CI group.

**Figure 2:** Comparison of measurement data between the CI group and the non-CI group: (a) course of DM; (b) time from onset to admission; (c) NIHSS score; (d) FBG, HbA1c, TG, TC, LDL-C, and HDL-C levels; and (e) TBIL, DBIL, Hcy, TSH, and Cys levels; (f): UA level.

**Figure 3:** ROC curves of peripheral blood miR-181c and miR-101 in the diagnosis of CI in patients with DM complicated with AS.

**Table 1:** Univariate analysis on the influencing factors of cognitive function in patients with DM complicated with AS [n(%)].

Index		CI group (*n* = 41)	Non-CI group (*n* = 29)	*χ * ^2^ value	*P -*Value
Gender (cases)	Male	25 (60.98)	18 (62.07)	0.810	0.368
	Female	16 (39.02)	11 (37.93)		
Age (year)	≤60	13 (31.71)	17 (58.62)	5.024	0.025
	>60	28 (68.29)	12 (41.38)		
Education level (cases)	Undergraduate and above	9 (21.95)	5 (17.24)	0.611	0.962
	Senior high school	19 (46.34)	14 (48.28)		
	Junior high school and below	13 (31.71)	10 (34.48)		
BMI (kg/m^2^)	≤24	24 (58.54)	16 (55.17)	18.290	0.919
	>24	17 (41.46)	13 (44.83)		
Combined underlying disease (cases)	Hypertension	12 (29.27)	7 (24.14)	0.226	0.634
	Coronary heart disease	9 (21.95)	6 (20.69)	0.016	0.899
Smoking history (cases)	No	26 (63.41)	18 (62.07)	0.013	0.909
	Yes	15 (36.59)	11 (37.93)		
History of drinking (cases)	No	29 (70.73)	19 (65.52)	0.214	0.643
	Yes	12 (29.27)	10 (34.48)		
AS location	Subtentorial	5 (12.20)	4 (13.79)	6.306	0.043
	Subcutaneous	23 (56.10)	23 (79.31)		
	Cortex	13 (31.70)	2 (6.90)		
Type of AS	Cerebral infarction	22 (53.66)	18 (62.07)	0.491	0.484
	Intracerebral hemorrhage	19 (46.34)	11 (37.93)		

**Table 2:** Assignments of study variables.

Index	Relevant factor	Definition and assignment	
*X*_1_	Age	≤60 years = 0	>60 years = 1
*X*_2_	DM course of disease	≤7.16 years = 0	>7.16 years = 1
*X*_3_	AS location	Subtentorial or subcutaneous = 0	, = 1
*X*_4_	Time from onset to admission	≤31.59 h = 0	>31.59 h = 1
*X*_5_	HbA1c	≤6.89% = 0	>6.89% = = 1
*X*_6_	TG	≤1.47mmoL/L = 0	>1.47mmoL/L = 1
*X*_7_	UA	≤279.45*μ*moL/L = 0	>279.45*μ*moL/L = 1
*X*_8_	Hcy	≤14.26*μ*moL/L = 0	>14.26*μ*moL/L = 1
*X*_9_	miR-181c	>0.91 = 0	≤0.91 = 1
X_10_	miR-101	>1.01 = 0	≤1.01 = 1

**Table 3:** Logistic regression analysis on the influencing factors of CI in patients with DM complicated with AS.

Index	*β*	SE	Wald *χ*^2^	OR	95%CI lower limit	95%CI upper limit	*P -*Value
Age	1.024	0.493	4.314	2.784	1.059	7.318	0.038
DM course of disease	0.977	0.536	3.322	2.656	0.929	7.596	0.069
AS location	0.992	0.438	5.130	2.697	1.143	6.363	0.024
Time from onset to admission	0.876	0.517	2.871	2.401	0.872	6.615	0.091
HbA1c	1.012	0.467	0.526	2.751	1.102	6.871	0.031
TG	0.983	0.522	3.546	2.672	0.976	7.319	0.056
UA	0.783	0.508	2.376	2.188	0.808	5.992	0.124
Hcy	0.826	0.514	2.582	2.284	0.834	6.255	0.109
miR-181c	1.015	0.473	4.605	2.759	1.092	6.973	0.032
miR-101	0.994	0.498	3.984	2.702	1.018	7.171	0.047

**Table 4:** ROC characteristics of peripheral blood miR-181c and miR-101 in the diagnosis of CI in patients with DM complicated with AS.

Index	AUC	Standard error	Sensitivity (%)	Specificity (%)	Cutoff value	95%CI	*P-value*
miR-181c	0.816	0.056	92.68	68.97	0.91	0.707∼0.925	<0.001
miR-101	0.783	0.057	73.17	82.76	1.01	0.671∼0.896	<0.001
Joint detection	0.865	0.045	73.17	89.66	—	0.777∼0.954	<0.001

## Data Availability

The data can be obtained from the author upon reasonable request.
